# Effect of Grading Rehabilitation Nursing Mode on Limb Function, Speech Rehabilitation, and Quality of Life of Stroke Patients

This article has been retracted.

**DOI:** 10.1155/2022/6956406

**Published:** 2022-08-02

**Authors:** Fen Qian, Yan Zhang, Yan Chen

**Affiliations:** ^1^Surgical Intensive Care Unit, Hai'an People's Hospital, Hai'an 226600, China; ^2^Department of Operating Room, Wuxi Second Hospital, Nanjing Medical University, Wuxi 214000, Jiangsu, China

## Abstract

**Objective:**

The aim of this study is to investigate the influence of grading rehabilitation nursing mode on limb function, speech function, and QOL of stroke patients.

**Methods:**

From January 2018 to April 2019, the stroke patients who received treatment in our hospital were selected as the study participants. Based on the random number table, they were assigned to CG (*n* = 60) and OG (*n* = 60). The routine rehabilitation nursing mode was used in the CG, and the grading rehabilitation nursing mode was used in the OG. The limb function, speech function, QOL, and nursing satisfaction were evaluated in both the groups, and the survival curve was analyzed after 12 months of follow-up.

**Results:**

The motor function of upper and lower limbs in OG was significantly higher than that in CG, and the total effective rate of speech function recovery in OG was 95.00%, which was obviously higher than 81.67% in CG (*P* < 0.05); the total QOL score in OG was (80.72 ± 7.15), which was significantly higher than (69.53 ± 6.42) in CG. The nursing satisfaction of the OG was higher (*P* < 0.05). The Kaplan–Meier curve analysis revealed that the difference of 12-month survival rate between CG and OG was statistically significant (*χ*^*2*^ = 4.710, *P*=0.030).

**Conclusion:**

The application of grading rehabilitation nursing mode in stroke patients can effectively facilitate the recovery of extremity function and speech function, ameliorate the QOL and nursing satisfaction of patients, reduce the death and disability of patients, and prolong the survival time of patients.

## 1. Introduction

Stroke is a disease in which the brain tissue is damaged due to a sudden rupture of blood vessels in the brain or blood cannot flow into the brain due to blockage of blood vessels. Studies have shown that the annual incidence of stroke in China has reached 2 million in recent years, and more than 70% of survived patients are left with varying degrees of limb dysfunction, which causes a heavy family financial burden and seriously affects the QOL of patients [1]. The main clinical manifestations are limb dysfunction (limb numbness and hemiplegia), language dysfunction (slurred words, inability to speak, etc.), and other dysfunctions. It enables the patient to lose the ability of daily living and affects the quality of life (QOL) of the patient [2]. Hence, the problem of how to improve the limb motor dysfunction of stroke patients, restore language function, and ameliorate the QOL of patients is a pressing topic and research focus in stroke rehabilitation nursing [3]. It is necessary to depend on comprehensive and standardized rehabilitation training to inhibit the development of the disease and promote the recovery of the patient's brain nerve function from the outside world due to the inability of brain function compensation on its own after a stroke.

Studies have proved that although the conventional nursing model has achieved certain results, it still can cause proportional disability because of the lack of scientificity, standardization, and poor prognosis [4]. Graded care refers to the fact that during the hospitalization of a patient, medical staff determine and implement different levels of care according to the patient's condition and self-care ability. There are four levels of graded care: special care, primary care, secondary care, and tertiary care. The graded nursing model allows nurses to know more about the treatment plan of loyal patients and promotes the expansion and improvement of nurses' clinical capabilities. By participating in the optimization and reconstruction of the department's workflow with doctors, mutual recognition and respect are promoted, and the job satisfaction of doctors and nurses is further improved, providing a strong guarantee for excellent service. The grading rehabilitation nursing model provides rehabilitation nursing care for patients from early nursing, rehabilitation nursing and later rehabilitation nursing, which can effectively ameliorate the neurological and cognitive functions of patients [5]. However, whether it is effective for limb function, linguistic function, and QOL still needs further study. Therefore, we mainly discuss the impact of grading rehabilitation nursing model on the limb function, language function, and QOL of stroke patients and provide reference for clinical reference.

## 2. Materials and Methods

### 2.1. General Information

From January 2018 to April 2019, we enrolled stroke patients who received treatment in our hospital as the research subjects.

#### 2.1.1. Inclusion Criteria

The inclusion criteria were as follows: (1) confirmed by CT, MRI, and other imaging examinations and met the diagnostic criteria for stroke (According to *Chinese guidelines for diagnosis and treatment of acute ischemic stroke (2014)*) [6]; (2) those with stroke for the first time; (3) those with limb dysfunction and language dysfunction; and (4) those volunteered to participate in the research and affixed an informed consent form.

#### 2.1.2. Exclusive Criteria

The exclusion criteria were as follows: (1) those with a history of circulatory and blood system diseases; (2) those with heart, liver, and kidney dysfunction; and (3) those with brain trauma, Alzheimer's disease, or communication disorders.

Finally, 120 patients were enrolled and assigned to CG (*n* = 60) and OG (*n* = 60) by the random number table method. All patients were 50–75 years old, and the course of disease was 1–15 days. This research was ratified by the ethics committee of Wuxi Second Hospital, Nanjing Medical University, Approval No. 779310. The basic data of the CG and OG were not statistically significant (*P* > 0.05). See Table 1 for details.

### 2.2. Methods

After admission, all patients received vital signs monitoring, infection prevention, nerve nutrition, microcirculation improvement, and intracranial pressure adjustment. The CG used conventional rehabilitation nursing model, including stroke-related knowledge education, rehabilitation training, and psychological nursing.

Based on the CG, the OG adopted a grading rehabilitation nursing model. The grade I early rehabilitation nursing care was implemented within 1 month after stroke treatment. The grade II rehabilitation nursing care was carried out within 2–3 months. The grade III late rehabilitation nursing care was conducted within 4–6 months [7]. The specific content is as follows. (1) Health knowledge education. We introduce the causes of stroke, the occurrence, and development of the disease, preventive measures and treatment methods to patients and their families. Then, we persuade and encourage patients to take part in rehabilitation treatment, appropriate self-training, or housework. We inform patients' family members of the correct nursing skills, handling method of complications, etc. [8]. (2) Limb function. Nursing staff should be gentle and instruct patients to stay in bed, turn over, and move. Patients in a stable condition are required to do the exercise such as raising arms over head, flexion and extension of lower limbs, swinging, etc., and are instructed to stand balance and walk with assistance. If the patient is in a good condition, they can perform daily behavior exercises such as simple washing, changing clothes, eating, and toileting [9]. (3) Diet nursing care (According to the *Dietary Guidelines for Stroke Patients (People's Republic of China Health Industry Standard Number: WS/T558-2017)*): We take a reasonable diet according to the dietary habits and condition of different patients. We choose low-salt, protein-rich soy products, eat more fresh vegetables and fruits, and other foods with high dietary fiber. It is forbidden to eat fried, irritating foods, and small meals are allowed. We provide intravenous nutritional support for patients who have difficulty eating. (4) Language function training: We instruct patients to exercise their mouth and tongue, bulging, blowing, tongue extension, tongue curling, etc.; we guide their pronunciation training, from the easy to the difficult and complicated, such as “ah”, “ah”, “b”, “p”, and other simple vocabulary, syllables, and sentences. Through multimedia channels such as watching TV programs, listening to the radio, reading books, and reading newspapers, patients are allowed to practice language expression and gradually improve their language ability; the patients are trained on hearing and vision to more comprehensively improve the patient's language function to ensure normal communication [10]. (5) Psychological nursing care. The recovery process after stroke is long, and the patient is prone to pessimism, anxiety, depression, irritability, and other negative psychology. Nursing staff need to communicate with patients and give psychological counseling to alleviate the patients' negative emotions; we use successful sample cases to further enhance their confidence and courage to overcome the disease. At the same time, family members should provide patients with a family support to actively cooperate with rehabilitation treatment.

### 2.3. Observation Indicators

The observation indicators were as follows: (1) The FuglMeyer motor assessment (FMA) scale was used to evaluate the limb function and movement of the two groups of patients [11], 33 items for the upper limb (sitting position), 17 items for the lower limb (supine position), each item 0–2 points; completely unable to perform or complete = 0 points, partially perform or complete = 1 point, fully perform or complete = 2 points. The upper limbs account for 66 points and lower limbs for 34 points, totaling 100 points. The higher the score, the better the limb function. (2) The speech function recovery of patients in both groups. Significantly effective: the speech function is basically restored, and normal communication with people is possible; effective: the speech function is gradually restored, and simple communication is possible; ineffective: the speech function is not improved and communication is not possible. (3) The FACT scale was applied to assess the QOL of patients in both groups after nursing [12], including mental function, physiological function, social function, cognitive function, and overall QOL score. The total score is 100 points, the higher the score, the better the function. (4) Nursing satisfaction score was classified as follows: very satisfied (80–100 points), generally satisfied (60–79 points), dissatisfied (<60 points), and the total score is 100 points. Satisfaction rating=(very satisfied + generally satisfied)/total number of cases *∗* 100%. (5) The Kaplan–Meier survival curve was applied to compare patients in both groups after being followed up for 12 months.

### 2.4. Statistical Methods

SPSS20.0 was applied to analyse the data. Quantitative data were represented by (*x* ± *s*), using *t*-test for comparison; qualitative data were expressed by (*n*%), using chi-squared test for comparison; the Kaplan–Meier curve was drawn. *P* < 0.05 represented a statistically significant difference.

## 3. Results

### 3.1. The Limb Motor Function of Patients in Both the Groups

After nursing, the motor function of upper and lower limbs of the OG was significantly better by contrast with the CG (*P* < 0.05), see Table 2 for details.

### 3.2. The Speech Function Recovery of Patients in Both the Groups before and after Nursing

The speech function recovery in OG after nursing showed higher total effective rate compared with the CG (95.00% vs 81.67%) (*P* < 0.05, Table 3).

### 3.3. The QOL of Patients in Both the Groups after Nursing

The OG demonstrated a higher total QOL score in comparison to ((80.72 ± 7.15) vs (69.53 ± 6.42)) (*P* < 0.05, Table 4).

### 3.4. Satisfaction after Nursing

The nursing satisfaction of the OG was 91.67% (55/60), which was obviously higher than 80.00% (48/60) of the CG (*P* < 0.05, Table 5).

### 3.5. Comparison of the 12-Month Survival Analysis

In both groups, patients were followed up for 12-month after being discharged from the hospital. In the CG, 8 patients died and 4 were censored, with a follow-up rate of 80.00%; In the OG, 4 patients died and 2 were censored, with a follow-up rate of 90.00%. The Kaplan–Meier curve analysis revealed that the difference of 12-month survival rate between CG and OG was statistically significant (*χ*^*2*^ = 4.710, *P*=0.030). See Figure 1.

## 4. Discussion

Stroke is a common acute cerebrovascular disease with extremely high morbidity, disability and mortality, and complicated pathogenesis [13]. The patients mainly manifest as limb, speech, and cognitive dysfunction. Traditional rehabilitation nursing training is usually carried out after the vital signs are stable, the nervous system symptoms are no longer aggravated, and the consciousness is clear (within 48 h) [14]. Nevertheless, there are drawbacks to the traditional model of care, which not only tends to ignore the psychological and social factors of the patient leading to conflict due to a lack of holistic care and a lack of communication and understanding. Nursing is also seen as a mechanical and repetitive task, where caregivers are unable to take initiative and be creative, and are prone to fatigue and boredom. As research progresses, some scholars believe that the earlier rehabilitation treatment is provided to patients, the better it is for the compensation and reconstruction of brain function [15]. If rehabilitation care training is provided within 12 hours after vital signs are stabilised, it can effectively alleviate patients' poor mental and depressive state and improve their daily living ability. Scientific and reasonable grading rehabilitation nursing care can facilitate the compensation and reorganization of the surrounding tissues and brain tissues of the healthy side or the affected side, accelerate the establishment of cerebral collateral circulation, facilitate the repair of damaged tissues and organs and the construction of central nervous system functions, and quickly restore the patient's limb function, language features and life ability [16].

In this study, the OG adopted a grading rehabilitation nursing model and the results showed that the upper and lower limb motor functions of the OG were obviously higher than those of the CG, and the total effective rate of speech function recovery after nursing was rather higher. It shows that the grading rehabilitation nursing model can facilitate the recovery of patients' extremity function and speech function. Under the guidance of rehabilitation medicine, this model involves early rehabilitation nursing and rehabilitation nursing care, which can ensure that patients access to scientific, comprehensive and standardized rehabilitation nursing, and repair the brain cell function of patients with ischemia and hypoxia, and reshape brain-computer functions, effectively promoting the recovery of limb motor function and daily life ability. This is consistent with relevant foreign research reports [17, 18]. The grading rehabilitation nursing model ensures the nursing outcomes from different grades. Grade I is carried out for the affected limbs to promote the blood circulation of the limbs and effectively prevent the deterioration of joint function. Grade II is carried out to restore the patient's speech function, daily self-care, and rehabilitation training to promote the recovery of the patient's cognitive function and neurological function. Grade III is carried out to supervise the patients, warning them to perform daily rehabilitation training, and regularly reviews. At the same time, psychological counseling for patients during nursing should be conducted, encouraging patients to cooperate with nursing intervention with a positive and optimistic attitude, establishing confidence in overcoming the disease, and striving for a speedy recovery [19].

Therefore, compared with the conventional rehabilitation nursing model implemented in the CG, the OG had higher total QOL score. At the meanwhile, the OG had better nursing satisfaction, indicating that the implementation of graded rehabilitation nursing can effectively promote the repair of neurological functions of stroke patients at all stages after the onset of stroke and improve the patients' recovery ability. The daily life of stroke patients and improve patient satisfaction. The Kaplan–Meier curve analysis showed that the comparison of 12-month survival rate between CG and OG was statistically significant (*χ*^*2*^ = 4.710, *P*=0.030). It shows that the application of grading rehabilitation nursing model for stroke patients has a good prognostic effect and can effectively ameliorate the clinical symptoms of patients, facilitate the recovery of patients' extremity function and speech function, increase the survival rate of patients, and reduce the mortality rate and the disability rate [20].

At present, many traditional Chinese medicines have played an important role in the treatment and prognosis of stroke patients, and they have been passed down because of their high efficiency, low cost, and convenience. The pathological factors of stroke in traditional Chinese medicine are the deficiency and the excess. The main pathological mechanism in the acute stage is blood stasis and phlegm turbidity, blocking the collaterals, and the methods of promoting blood circulation and removing blood stasis and fragrant opening are commonly used. Its risk factors include age, hypertension, diabetes, hyperlipidemia, and so on. Prevention of stroke requires timely control of the primary disease, improvement of unhealthy lifestyles and habits, followed by initiation of secondary prevention therapy, which mainly includes blood pressure control, antipolymerization and lipid regulation plus plaque stabilization; moreover, combination of the three methods can reduce the risk of stroke. 80% incidence [21, 22]. Chinese medicine emphasizes on stroke care: maintain emotional well-being and reduce adverse stimulation; keep the room sunny and ventilated; eat more light, digestible, high-quality protein-rich foods; carry out traditional Chinese medicine special care, such as cupping, acupuncture and traditional Chinese medicine fumigation; often observe the vital signs and state of consciousness of the patients in the acute stage, and pay attention to the nursing of the second bowel movement [23, 24]. In the future, we can innovate on the existing basis of traditional Chinese medicine and combine western medicine methods to develop new methods of diagnosis and treatment.

Inevitably, there is some chance in the experiment that may cause errors. For this study, our sample size was small and there may be regional differences within a certain range. Then again, this is a single-center clinical study. The rehabilitation of stroke patients is a long-term process, and we need regular follow-up in the later period to verify the more profound impact of graded rehabilitation care on the long-term quality of life of patients.

In summary, the grading rehabilitation nursing model for stroke patients can effectively promote the recovery of the patient's limb function and speech function, while improving the patient's QOL and nursing satisfaction, reducing the death and disability of the patient, and prolonging the survival time.

## Figures and Tables

**Figure 1:** Kaplan–Meier survival curve at 12 months follow-up in two groups. Patients in both groups were followed up for 12 months after discharge. There were 8 deaths and 4 deletions in CG, with a follow-up rate of 80.00%; 4 deaths and 2 tail amputations in OG, with a follow-up rate of 90.00%. The Kaplan–Meier curve analysis showed a statistically significant difference in 12-month survival rates between CG and OG.

**Table 1:** Comparison of general data (n (%), (‾*x* ± *s*)).

Groups	*n*	*Sex*		*Stroke types*		Average age (year)	Average disease course (d)
		Male	Female	Ischemic	Hemorrhagic		
Control group	60	33	27	42	18	61.24 ± 4.53	8.79 ± 2.06
Observation group	60	34	26	43	17	62.48 ± 4.76	8.64 ± 2.13
*χ * ^*2*^ * /t*		0.034		0.040		1.462	0.391
*P*		0.854		0.841		0.146	0.695

**Table 2:** The limb motor function of the two groups of patients (‾*x* ± *s*, point).

Groups	*Upper limb*		*Lower limb*	
	Before nursing	After nursing	Before nursing	After nursing
Control group	37.35 ± 6.38	46.12 ± 3.26	18.43 ± 4.05	22.58 ± 2.14
Observation group	37.86 ± 6.29	59.45 ± 3.17	18.74 ± 4.26	28.54 ± 2.83
*t*	0.440	22.710	0.408	13.010
*P*	0.660	<0.001	0.683	<0.001

**Table 3:** The speech function recovery of the two groups of patients (n (%)).

Groups	*n*	Markedly effective	Effective	Ineffective	Total effective rate
Control group	60	28 (46.67)	21 (35.00)	11 (18.33)	49 (81.67)
Observation group	60	33 (55.00)	24 (40.00)	3 (5.00)	57 (95.00)
*χ * ^*2*^					5.175
*P*					0.023

**Table 4:** Comparison of quality of life (‾*x* ± *s*, point).

Groups	*n*	Mental function	Physiological function	Social function	Cognitive function	Overall quality of life score
Control group	60	66.47 ± 5.19	63.75 ± 5.43	62.84 ± 4.67	65.36 ± 4.25	69.53 ± 6.42
Observation group	60	72.56 ± 6.08	76.49 ± 5.72	68.47 ± 4.38	78.59 ± 5.13	80.72 ± 7.15
*T*		5.901	12.510	6.811	15.380	9.020
*P*		<0.001	<0.001	<0.001	<0.000	<0.001

**Table 5:** Comparison of satisfaction (n (%)).

Groups	*n*	Satisfied	Generally satisfied	Dissatisfied	Satisfaction rating
Control group	60	27 (45.00)	21 (35.00)	12 (20.00)	48 (80.00)
Observation group	60	32 (53.34)	23 (38.33)	5 (8.33)	55 (91.67)
*χ * ^*2*^					5.316
*P*					0.021

## Data Availability

All data generated or analysed during this study are included in this published article.
